The article "Open versus endoscopic carpal tunnel release: a systematic review and meta-analysis of randomized controlled trials" was published in 2020. Journal: BMC Musculoskelet Disord.

# Open versus endoscopic carpal tunnel release: a systematic review and meta-analysis of randomized controlled trials

**DOI:** 10.1186/s12891-020-03306-1

**Published:** 2020-04-27

**Authors:** Yueying Li, Wenqi Luo, Guangzhi Wu, Shusen Cui, Zhan Zhang, Xiaosong Gu

**Affiliations:** 1 Department of Hand Surgery, China-Japan Union Hospital of Jilin University, No. 126 Xiantai Street, Changchun, Jilin 130033 P.R. China; 2 Department of Orthopedics, China-Japan Union Hospital of Jilin University, No. 126 Xiantai Street, Changchun, Jilin 130033 P.R. China

**Keywords:** Carpal tunnel syndrome, Complications, Endoscopic carpal tunnel release, Meta-analysis, Open carpal tunnel release, Randomized controlled trial

## Abstract

**Background:**

Endoscopic carpal tunnel release (ECTR) and open carpal tunnel release (OCTR) both have advantages and disadvantages for the treatment of carpal tunnel syndrome (CTS). We compared the effectiveness and safety of ECTR and OCTR based on evidence from a high-level randomized controlled trial.

**Methods:**

We comprehensively searched PubMed, EMBASE, Cochrane Library, Web of Science, and Medline to identify relevant articles published until August 2019. Data regarding operative time, grip strength, Boston Carpal Tunnel Questionnaire scores, digital sensation, patient satisfaction, key pinch strength, return to work time, and complications were extracted and compared. All mean differences (MD) and odds ratios (OR) were expressed as ECTR relative to OCTR.

**Results:**

Our meta-analysis contained twenty-eight studies. ECTR was associated with significantly higher satisfaction rates (MD, 3.13; 95% confidence interval [CI], 1.43 to 4.82; *P* = 0.0003), greater key pinch strengths (MD, 0.79 kg; 95% CI, 0.27 to 1.32; *P* = 0.003), earlier return to work times (MD, − 7.25 days; 95% CI, − 14.31 to − 0.19; *P* = 0.04), higher transient nerve injury rates (OR, 4.87; 95% CI, 1.37 to 17.25; *P* = 0.01), and a lower incidence of scar-related complications (OR, 0.20; 95% CI, 0.07 to 0.59; *P* = 0.004). The permanent nerve injury showed no significant differences between the two methods (OR, 1.93; 95% CI, 0.58 to 6.40; *P* = 0.28).

**Conclusions:**

Overall, evidence from randomized controlled trials indicates that ECTR results in better recovery of daily life functions compared to OCTR, as revealed by higher satisfaction rates, greater key pinch strengths, earlier return to work times, and fewer scar-related complications. Our findings suggest that patients with CTS can be effectively managed with ECTR.

## Background

Carpal tunnel syndrome (CTS), known as compressive median mononeuropathy at the wrist, causes tingling, numbness, and pain along the radial side of the hand [1]. The reported estimates for its annual prevalence range from 0.18 to 5% [2–5]. CTS can be treated surgically or non-surgically; however, non-surgical management that involves wrist splinting, corticosteroid injections, and physiotherapy, is preferred over surgical management for mild and moderate CTS [6, 7]. Surgical treatments for CTS, including the open carpal tunnel release (OCTR) and endoscopic carpal tunnel release (ECTR) approach, are generally reserved for patients with severe symptoms or those who experienced conservative treatment failure [8, 9].

The article "Open versus endoscopic carpal tunnel release: a systematic review and meta-analysis of randomized controlled trials" was published in 2020. Journal: BMC Musculoskelet Disord.

OCTR is a well-established surgical treatment for CTS [10]. However, it is associated with potential complications such as persistent weakness, pillar pain, formation of hypertrophic scars in the incisions that cross the wrist, scar tenderness, slow recovery, and a higher incidence of persistent pain [11]. In an attempt to avoid these complications, Chow [12] and Okutsu et al. [13] were the first to report the use of ECTR for the treatment of CTS in the English literature in 1989. This method allows for smaller skin incisions and better esthetic results than OCTR [1, 14, 15]. Nevertheless, ECTR is technically difficult, time consuming, and associated with incomplete transverse carpal ligament release and neurovascular injury [16–20]. Several meta-analyses have compared various measures of effectiveness and safety between ECTR and OCTR [15, 21–23]. However, these investigations failed to separate subgroups according to different follow-up times and utilized limited evaluations of patient outcomes; therefore, it is not clear which approach is associated with better clinical results [24, 25].

Therefore, we carried out a meta-analysis to compare the safety and availability between ECTR and OCTR according to randomized controlled trial (RCT) evidence. Specifically, we sought to determine if ECTR was superior to OCTR in terms of patient satisfaction, functional recovery, and complications.

## Methods

### Literature search

The Preferred Reporting Items for Systematic Reviews and Meta-Analyses (PRISMA) trial flow shows the inclusion process for the RCTs in the meta-analysis [26]. Two authors respectively used the following computerized bibliographic databases: PubMed, EMBASE, Cochrane Library, Web of Science, and Medline databases to search for relevant publications. Publications from the inception of each database to August 10, 2019 were searched. The keywords used in the searches were “carpal tunnel” plus “open incision” and “carpal tunnel” plus “endoscopic.” We also manually scanned the reference lists to identify other relevant studies, that were discovered using these search terms.

The article "Open versus endoscopic carpal tunnel release: a systematic review and meta-analysis of randomized controlled trials" was published in 2020. Journal: BMC Musculoskelet Disord.

### Eligibility criteria

A study was included if it was an RCT that compared OCTR and ECTR. The exclusion criteria were as follows: 1) descriptive or graphic outcomes with no standard deviation values, 2) studies that included modification surgery, 3) studies that did not coverage the follow-up time, 4) studies that only recorded limited qualitative findings, 5) studies published in a language other than English or Chinese, and 6) technique articles, abstracts, and nontherapeutic studies. Finally, two investigators independently reviewed all selected studies for inclusion.

### Data abstraction

Two authors extracted valuable data from the included studies respectively. When data heterogeneity is present, it must be resolved by containing a third author until data heterogeneity was reached a consensus for all items.

The extracted data included publication year, region, sample capacity, intervention, follow-up interval, and outcomes in eligible studies. Plot-digitizing software (Plot Digitizer Version 2.6.4; Joseph Huwaldt and Scott Steinhorst, http://www.plot-digitizer.com-about.com/) was used to quantify the data only recorded graphically. The pooled analysis outcome parameters were as follows: operation duration; scores on several clinical indexes, including the Boston Carpal Tunnel Questionnaire Symptom Severity Scale (BCTQ-S), Boston Carpal Tunnel Questionnaire Functional Status Scale (BCTQ-F), Two-point Discrimination test, and Semmes-Weinstein monofilament test; grip strength; key pinch strength; time to return to work (RTW); patients’ subjective ratings of their satisfaction with symptom improvement following CTS release based on a scale of 0 to 100 points; and postoperative complications.

### Validity assessment

The level of evidence was assessed by the Grading of Recommendations Assessment, Development, and Evaluation (GRADE) guidelines [27]. At least two authors respectively evaluated the risk of bias, and disagreements were discussed until a consensus was reached.

### Statistical analysis

Continuous data were analyzed through the inverse-variance statistical and method and mean difference (MD) and 95% confidence intervals (CIs) were reported. Dichotomous data were analyzed through the Mantel-Haenszel statistical method and odds ratio (OR) and 95% CI were reported. All MD and OR values were collected and collated using the results from OCTR as the reference values. In addition, χ^2^ and I^2^ tests were percentage of total variation that were used to assess statistical heterogeneity. When the *P* value from the χ^2^ test was < 0.10 or when the I^2^ value > 50% significant heterogeneity was indicated, the possible sources of heterogeneity were examined. Pooled result of the outcome was assessed by random-effects model; otherwise, a fixed-effects model was used. All tests were two-tailed, and *P* < 0.05 were considered statistically significant. The funnel plot method and Egger’s test were utilized to evaluate the publication bias. Review Manager (version 5.3; The Nordic Cochrane Centre, Cochrane Collaboration, Copenhagen, Denmark) was used to further analyze the data.

The article "Open versus endoscopic carpal tunnel release: a systematic review and meta-analysis of randomized controlled trials" was published in 2020. Journal: BMC Musculoskelet Disord.

## Results

### Studies selection and characteristics

Figure 1 summarizes the screening process of the identified articles in the final analysis. In the aggregate 5654 articles were confirmed from PubMed (*n* = 1416), EMBASE (*n* = 1755), Cochrane Library (*n* = 248), Web of Science (*n* = 1130), Medline (*n* = 1105), and reference lists (*n* = 0). After eliminated duplicates, 2248 articles remained. Reviews of the titles and abstracts decreased the articles to 103, finally this number reduced to 28 articles included in the meta-analysis after a more detailed review. Twenty-seven articles were published in English and one was published in Chinese. The included article characteristics are summed up in Table 1.

**Fig. 1:** Flow diagram of the study selection process

**Table 1:** Study characteristics of the randomized controlled trials included in the meta-analysis

Author	Year	Region	Groups, sample sizes, and techniques	Follow-up interval	Outcomes
Agee et al. [28]	1992	US	OCTR (*n* = 65): conventional release ECTR (*n* = 82): one-portal (2 cm)	1, 2, 3, 6, 9, 13, 26 week(s)	Return of hand use for ADL, time to RTW, grip strength, pinch strength, lateral/key and pulp strength, SW monofilament test, Phalen’s wrist flexion test, Tinel’s test, scar tenderness, radial and ulnar pillar tenderness, record of medication use, complications
Atroshi et al. [9]	2006	Sweden	OCTR (*n* = 65): 4 cm ECTR (*n* = 63): two-portal (1 cm)	3, 6 weeks; 3, 12 months	Pain, time to RTW, BCTQ-S, BCTQ-F, SF-12, sensation, grip strength, key pinch strength, DL, quality of life, SW monofilament test, 2PD test, complications
Atroshi et al. [29]	2009	Sweden	OCTR (*n* = 63): 4 cm ECTR (*n* = 63): two-portal (1 cm)	1, 5 year(s)	Operative time, satisfaction rating, symptom relief, BCTQ-S, BCTQ-F, pain score, complications
Atroshi et al. [25]	2015	Sweden	OCTR (*n* = 61): 4 cm ECTR (*n* = 63): two-portal (1 cm)	1, 11–16 year(s)	BCTQ-S, BCTQ-F, pain score, numbness and tingling, satisfaction score, quick DASH, pain scale, complications
Aslani et al. [30]	2012	Iran	OCTR (*n* = 36): conventional release OCTR (*n* = 28): mini-incision ECTR (*n* = 32): two-portal (length NR)	4 weeks; 4 months	Numbness, nocturnal pain, wrist pain, weakness and stiffness, Tinel’s test, Phalen’s wrist flexion test, EMG, NCV, strength to grasp, time to RTW and ADL, satisfaction rating, operative time, complications
Brown et al. [31]	1993	US	OCTR (*n* = 82): conventional release ECTR (*n* = 78): two-portal (2 cm)	3, 6, 12 weeks	2PD test, SW monofilament test, APB strength, thenar atrophy, grip strength, key pinch strength, pain, numbness, paresthesia, weakness, Tinel’s test, Phalen’s wrist flexion test, interstitial carpal tunnel pressure, satisfaction rating, time to RTW, rate of ADL impairment, ADL score, operative time, hospital cost, complications
Dumontier et al. [32]	1995	France	OCTR (*n* = 40): conventional release ECTR (*n* = 56): two-portal (Chow [12])	2 weeks; 1, 3, 6 month(s)	Paresthesia, pain, time to RTW, grip strength, finger mobility, complications
Ejiri et al. [33]	2012	Japan	OCTR (*n* = 50): 3 cm vertical incision ECTR (*n* = 50): one-portal (Okutsu et al. [13])	1, 3 month(s)	Paresthesia, nighttime pain, impairment of ADL, APB-DL, SW monofilament test, 2PD test, grip strength, pinch strength, key pinch strength, complications
Erdmann [34]	1994	UK	OCTR (*n* = 52): NR (short length) ECTR (*n* = 53): two-portal (Chow [12])	1, 2 week(s); 1, 3, 6 month(s); 1 year	Grip and pinch strength, time to normal grip strength, time to normal pinch strength, time to RTW, ADL, time to relief of symptoms, median nerve motor and sensory DL, VAS pain score, complications
Ferdinand and MacLean [35]	2002	UK	OCTR (*n* = 25): NR ECTR (*n* = 25): one-portal	6, 12, 26 weeks; 13 months	VAS scores (numbness, pain, and paresthesia), ADL, return to full activities, time to RTW, thenar muscle strength, lateral pinch strength, grip strength, wrist and finger movement, 2PD test, Jebson score, operative time, satisfaction rating, complications
Gümüştaş et al. [36]	2015	Turkey	OCTR (*n* = 20): NR (Taleisnik [37]) ECTR (*n* = 21): two-portal (Chow [12])	6 months	BCTQ-S, BCTQ-F, median nerve motor DL, CMAP, SCV, sensory nerve action potential, complications
Jacobson and Rahme [38]	1996	Sweden	OCTR (*n* = 16): conventional release ECTR (*n* = 16): two-portal (Chow [12])	2, 6, 24 weeks	Symptom relief, total number of analgesics, 2PD test, time to RTW, nerve conduction test, complications
Kang et al. [39]	2013	South Korea	OCTR (*n* = 52): mini-incision (1.5 cm) ECTR (*n* = 52): one-portal (Agee et al. [28])	3 months	BCTQ-S, BCTQ-F, DASH, complications
Larsen et al. [40]	2013	Denmark	OCTR (*n* = 30): classic incision, 7 cm OCTR (*n* = 30): short incision, 3 cm ECTR (*n* = 30): one-portal (Menon [41])	1, 2, 3, 6, 12, 24 week(s)	VAS (pain), grip strength, range of motion, pillar pain, VAS (paresthesia), time to RTW, complications
Macdermid et al. [42]	2003	Canada	OCTR (*n* = 32): conventional release ECTR (*n* = 91): two-portal (Chow [12])	1, 6, 12 week(s)	Time to RTW, McGill pain questionnaire, key pinch strength, tripod pinch strength, grip strength, symptom severity score (Likert score), sensory threshold, self-report scale, SF-36, complications
Mackenzie et al. [43]	2000	US	OCTR (*n* = 14): 2.5 cm palmar incision ECTR (*n* = 22): one-portal (Agee et al. [28])	1, 2, 4 week(s)	Grip strength, pinch strength, BCTQ-S, BCTQ-F, complications
Martínez et al. [24]	2019	Spain	OCTR (*n* = 52): 1 cm mini-incision ECTR (*n* = 35): one-portal (Menon [41])	1 week; 1, 6, 12 month(s)	Grip strength, pinch strength, VAS pain score, satisfaction questionnaire, complications
Michelotti et al. [44]	2014	US	OCTR (*n* = 25): 3 cm palmar incision ECTR (*n* = 25): one-portal (Agee et al. [28], 1.5 cm)	2, 4, 8, 12, 24 weeks	2PD test, SW monofilament test, thenar strength, grip strength, BCTQ-S, BCTQ-F, satisfaction rating, complications
Michelotti et al. [45]	2018	US	OCTR (*n* = 30): 3 cm palmar incision ECTR (*n* = 30): one-portal (Agee et al. [28], 1.5 to 2 cm)	2, 4, 8, 12, 24 weeks	VAS pain score, 2PD test, SW monofilament test, thenar strength, grip strength, BCTQ-S, BCTQ-F, satisfaction rating, complications
Oh et al. [46]	2017	South Korea	OCTR (*n* = 32): mini-incision (1.5 cm) ECTR (*n* = 35): one-portal (Agee et al. [28], 1.5 cm)	24 weeks	BCTQ-S, BCTQ-F, DASH, CSA, CSA-I, CSA-M, CSA-O, flattening ratio, complications
Rab et al. [47]	2006	Austria	OCTR (*n* = 10): two mini-incisions ECTR (*n* = 10): two-portal (Chow [12])	2, 4, 6, 12 weeks; 6, 12 months	VAS pain score, grip strength, pinch strength, key pinch strength, ADL, BCTQ-S, BCTQ-F, 2PD, DL, NCV, complications
Saw et al. [48]	2003	UK	OCTR (*n* = 42): 2 cm palmar incision ECTR (*n* = 43): one-portal (Agee et al. [28])	1, 3, 6, 12 week(s)	BCTQ-S, BCTQ-F, grip strength, VAS pain score, time to RTW, operation time, complications
Sennwald and Benedetti [49]	1995	Switzerland	OCTR (*n* = 22): Sennwald incision ECTR (*n* = 25): one-portal (Agee et al. [28], 2–3 cm)	4, 8, 12 weeks	Grip strength, key pinch strength, time to RTW, complications
Tian et al. [50]	2007	China	OCTR (*n* = 36): S-shaped incision ECTR (*n* = 34): one-portal (Okutsu et al. [13], 1 cm)	2 years	Symptom improvement, operation time, hospital stay time, time to RTW, 2PD test, grip strength, scar tenderness, complications
Trumble et al. [51]	2002	US	OCTR (*n* = 95): palmar incision (3 ~ 4 cm) ECTR (*n* = 97): one-portal (Agee et al. [28], 1 cm)	2, 4, 8, 12, 26, 52 weeks	BCTQ-S, BCTQ-F, 2PD test, satisfaction rating, grip strength, pinch strength (key pinch, three-jaw), hand dexterity, time to RTW, thenar atrophy, strength of APB, complications
Wong et al. [52]	2003	Hong Kong	OCTR (*n* = 30): mini-incision ECTR (*n* = 30): two-portal (Chow [12])	2, 4, 8, 16 weeks; 6, 12 months	VAS pain score, grip strength, pinch strength, 2PD test, operation time, symptom relief, incision length, complications
Zhang et al. [53]	2016	China	OCTR (*n* = 72): double small incision OCTR (*n* = 65): standard incision (5–7 cm) ECTR (*n* = 69): two-portal (Chow [12])	3 years	BCTQ-S, BCTQ-F, patient satisfaction, VAS pain score, cylindrical strength, lateral strength, pinch strength, grip strength, time to RTW, 2PD test, SW monofilament test, hospital cost, complications
Zhao et al. [54]	2004	China	OCTR (*n* = 21): S-shaped incision ECTR (*n* = 26): one-portal (Okutsu et al. [13], 1 cm)	2 years	EMG, operation time, hospital stay time, 2PD test, time to RTW, complications

*2PD* Two-point Discrimination, *ADL* activities of daily living, *APB* abductor pollicis brevis, *BCTQ-F* Boston Carpal Tunnel Questionnaire Functional Status Scale, *BCTQ-S* Boston Carpal Tunnel Questionnaire Symptom Severity Scale, *CMAP* compound muscle action potential, *CSA* cross-sectional area, *CSA-I* inlet at the distal wrist crease level, *CSA-M* the middle of the tunnel at the level of the pisiform, *CSA-O* the tunnel outlet at the level of the hamate hook, *DASH* Disability of Arm, Shoulder, and Hand Questionnaire, *DL* distal latency, *ECTR* endoscopic carpal tunnel release, *EMG* electromyography, *NCV* nerve conduction velocity, *NR* not reported, *OCTR* open carpal tunnel release, *RTW* return to work, *SCV* sensory conduction velocity, *SF-12* 12-Item Short Form Health Survey, *SF-36* 36-Item Short Form Health Survey, *SW* Semmes-Weinstein, *UK* United Kingdom, *US* United States, *VAS* Visual Analog Scale

The article "Open versus endoscopic carpal tunnel release: a systematic review and meta-analysis of randomized controlled trials" was published in 2020. Journal: BMC Musculoskelet Disord.

### Quality assessment

In line with GRADE guidelines, 19 RCTs reported adequate methods for selection bias of random sequence generation. Only 8 RCTs had low risks of blinding of outcome assessment for results. The majority of RCTs (25/28) had risk of performance bias. Incomplete outcome data was judged as low risk for 22 RCTs. All RCTs were at a low risk of reporting bias (Fig. 2).

**Fig. 2:** Risk of bias assessment for included randomized controlled trials

### Results of meta-analysis

There were no significant differences in the operative time (MD, − 5.81 min; 95% CI, − 17.85 to 6.23; *P* = 0.34; *n* = 261; random-effects model, I^2^ = 99%; *P* < 0.00001; Fig. 3) [35, 39, 52, 54], grip strength at 3 months post-surgery (MD, 1.99 kg; 95% CI, − 0.43 to 4.42; *P* = 0.11; *n* = 297; fixed-effects model, I^2^ = 0%; *P* = 0.79; Fig. 4) [9, 31], BCTQ-S score at 1 year post-surgery (MD, 0.15; 95% CI, − 0.04 to 0.35; *P* = 0.13; *n* = 592; random-effects model, I^2^ = 92%; *P* < 0.00001; Fig. 5) [25, 51, 53], and BCTQ-F score at 1 year post-surgery (MD, 0.17; 95% CI, − 0.02 to 0.36; *P* = 0.08; *n* = 592; random-effects model, I^2^ = 91%; *P* < 0.00001; Fig. 6) [25, 51, 53] between the ECTR and OCTR groups. Similarly, there were no differences in digital sensation, including the Semmes-Weinstein monofilament test score at 3 months post-surgery (MD, 0.06; 95% CI, − 0.09 to 0.21; *P* = 0.43; *n* = 297; fixed-effects model, I^2^ = 0%; *P* = 0.65; Fig. 7) [9, 31] and Two-point Discrimination test score at 1 year post-surgery (MD, − 0.16; 95% CI, − 0.45 to 0.12; *P* = 0.26; *n* = 402; fixed-effects model, I^2^ = 35%; *P* = 0.20; Fig. 8) [50, 52, 53], between the two groups.

**Fig. 3:** Comparison of operative time between patients who underwent ECTR and those who underwent OCTR. OCTR, open carpal tunnel release; ECTR, endoscopic carpal tunnel release; SD, standard deviation; IV, inverse-variance; CI, confidence interval; df, degrees of freedom

**Fig. 4:** Comparison of grip strength between patients who underwent ECTR and those who underwent OCTR. OCTR, open carpal tunnel release; ECTR, endoscopic carpal tunnel release; SD, standard deviation; IV, inverse-variance; CI, confidence interval; df, degrees of freedom

**Fig. 5:** Comparison of the Boston Carpal Tunnel Questionnaire Symptom Severity Scale (BCTQ-S) score between patients who underwent ECTR and those who underwent OCTR. OCTR, open carpal tunnel release; ECTR, endoscopic carpal tunnel release; SD, standard deviation; IV, inverse-variance; CI, confidence interval; df, degrees of freedom

**Fig. 6:** Comparison of the Boston Carpal Tunnel Questionnaire Functional Status Scale (BCTQ-F) score between patients who underwent ECTR and those who underwent OCTR. OCTR, open carpal tunnel release; ECTR, endoscopic carpal tunnel release; SD, standard deviation; IV, inverse-variance; CI, confidence interval; df, degrees of freedom

**Fig. 7:** Forest plots showing the standardized mean difference for the Semmes-Weinstein (SW) monofilament test between patients who underwent ECTR and those who underwent OCTR. ECTR, endoscopic carpal tunnel release; OCTR, open carpal tunnel release; IV, inverse-variance; CI, confidence interval; df, degrees of freedom

**Fig. 8:** Forest plots showing the standardized mean difference for the Two-point Discrimination (2PD) test between patients who underwent ECTR and those who underwent OCTR. ECTR, endoscopic carpal tunnel release; OCTR, open carpal tunnel release; IV, inverse-variance; CI, confidence interval; df, degrees of freedom

The article "Open versus endoscopic carpal tunnel release: a systematic review and meta-analysis of randomized controlled trials" was published in 2020. Journal: BMC Musculoskelet Disord.

#### Satisfaction rate

The overall level of satisfaction with the outcome was based on a scale of 0 to 100 points. Two articles provided comparative data on the satisfaction rate [31, 53]. A portion of the data from Zhang et al. [53] reported a satisfaction rate of up to 90%, with high heterogeneity; therefore, some of the satisfaction data from that study were eliminated from the present meta-analysis. The pooled data of the two articles showed that the satisfaction rate was significantly higher in the ECTR group than that in the OCTR group (MD, 3.13; 95% CI, 1.43 to 4.82; *P* = 0.0003; *n* = 303; I^2^ = 0%; *P* = 0.57) [31, 53], and the clinical heterogeneity I^2^ was null (Fig. 9).

**Fig. 9:** Comparison of overall satisfaction ratings after CTS release between patients who underwent ECTR and those who underwent OCTR. OCTR, open carpal tunnel release; ECTR, endoscopic carpal tunnel release; SD, standard deviation; IV, inverse-variance; CI, confidence interval; df, degrees of freedom

#### Key pinch strength

The pooled data showed that the key pinch strength of patients who were treated with ECTR was significantly greater than the key pinch strength of patients who were treated with OCTR at 3-months post-surgery (MD, 0.79 kg; 95% CI, 0.27 to 1.32; *P* = 0.003; *n* = 297; fixed-effects model, I^2^ = 0%; *P* = 0.70) [9, 31] (Fig. 10).

**Fig. 10:** Comparison of key pinch strength between patients who underwent ECTR and those who underwent OCTR. OCTR, open carpal tunnel release; ECTR, endoscopic carpal tunnel release; SD, standard deviation; IV, inverse-variance; CI, confidence interval; df, degrees of freedom

#### RTW

Four studies [30, 38, 48, 54] evaluated the time needed to return to work for patients who underwent CTS. The pooled data showed that the RTW times were significantly faster in patients in the ECTR group than those in the OCTR group (MD, − 7.25 days; 95% CI, − 14.31 to − 0.19; *P* = 0.04; *n* = 357; random-effects model, I^2^ = 98%; *P* < 0.00001) (Fig. 11); however, divergences between studies resulted in large between-study heterogeneity.

**Fig. 11:** Comparison of the time to return to work (RTW) between patients who underwent ECTR and those who underwent OCTR. OCTR, open carpal tunnel release; ECTR, endoscopic carpal tunnel release; SD, standard deviation; IV, inverse-variance; CI, confidence interval; df, degrees of freedom

#### Complications

Twenty-five studies [9, 24, 28, 30–36, 38–40, 42, 43, 45–54] included complete complication rate data and were included in the pooled analysis of overall complications. There were no significant differences between all complications rates (OR, 1.06; 95% CI, 0.69 to 1.64; *P* = 0.78; *n* = 2320; fixed-effects model, I^2^ = 16%; *P* = 0.27) (Fig. 12). The rates of transient nerve injury were higher in patients who underwent ECTR than those in patients who underwent OCTR (OR, 4.87; 95% CI, 1.37 to 17.25; *P* = 0.01; *n* = 2320; fixed-effects model, I^2^ = 0%; *P* = 0.98) (Fig. 13); however, the studies provided evidence that the presence of permanent nerve injury was not significantly different between the two groups (OR, 1.93; 95% CI, 0.58 to 6.40; *P* = 0.28; *n* = 2320; fixed-effects model, I^2^ = 29%; *P* = 0.24) (Fig. 14). The rates of scar-related complications (scar hypertrophy, scar hyperesthesia, scar pain) were lower in patients who underwent ECTR than those in patients who underwent OCTR (OR, 0.20; 95% CI, 0.07 to 0.59; *P* = 0.004; *n* = 2320; fixed-effects model, I^2^ = 0%; *P* = 0.90) (Fig. 15). Other complications, such as hematoma, wound infection, superficial palmar arch injury, persistent symptoms, pillar pain, reflex sympathetic dystrophy, and tendon injury, different were not significantly between the two groups. All outcome variables are summed up and displayed in Table 2.

The article "Open versus endoscopic carpal tunnel release: a systematic review and meta-analysis of randomized controlled trials" was published in 2020. Journal: BMC Musculoskelet Disord.

**Fig. 12:** Comparison of all complications between patients who underwent ECTR and those who underwent OCTR. ECTR, endoscopic carpal tunnel release; OCTR, open carpal tunnel release; M-H, Mantel-Haenszel; CI, confidence interval; df, degrees of freedom

**Fig. 13:** Comparison of transient nerve injury between patients who underwent ECTR and those who underwent OCTR. ECTR, endoscopic carpal tunnel release; OCTR, open carpal tunnel release; M-H, Mantel-Haenszel; CI, confidence interval; df, degrees of freedom

**Fig. 14:** Comparison of permanent nerve injury between patients who underwent ECTR and those who underwent OCTR. ECTR, endoscopic carpal tunnel release; OCTR, open carpal tunnel release; M-H, Mantel-Haenszel; CI, confidence interval; df, degrees of freedom

**Fig. 15:** Comparison of scar-related complications between patients who underwent ECTR and those who underwent OCTR. ECTR, endoscopic carpal tunnel release; OCTR, open carpal tunnel release; M-H, Mantel-Haenszel; CI, confidence interval; df, degrees of freedom

**Table 2:** Summary estimates of outcome variables in the current study

Outcome	No. of studies	Heterogeneity I^2a^ (%)	Pooled odds ratio^b^	Mean difference^c^	95% confidence interval (lower bound)	95% confidence interval (upper bound)
Operative time	4	99	NA	−5.81	−17.85	6.23
Grip strength	2	0	NA	1.99	−0.43	4.42
BCTQ-S score	3	92	NA	0.15	−0.04	0.35
BCTQ-F score	3	91	NA	0.17	−0.02	0.36
SW monofilament test score	2	0	NA	0.06	−0.09	0.21
2PD test score	3	35	NA	−0.16	−0.45	0.12
Satisfaction rate	2	0	NA	3.13	1.43	4.82
Key pinch strength	2	0	NA	0.79	0.27	1.32
Return to work	4	98	NA	−7.25	−14.31	−0.19
Complications	25	16	1.06	NA	0.69	1.64
Transient nerve injury	25	0	4.87	NA	1.37	17.25
Permanent nerve injury	25	29	1.93	NA	0.58	6.4
Scar-related complications	25	0	0.2	NA	0.07	0.59
Hematoma	25	0	1.60	NA	0.36	7.16
Wound infection	25	0	0.53	NA	0.15	1.97
Superficial palmar arch injury	25	NA	3.07	NA	0.12	76.48
Persistent symptoms	25	0	2.17	NA	0.85	5.55
Pillar pain	25	35	0.95	NA	0.32	2.82
Reflex sympathetic dystrophy	25	0	0.40	NA	0.10	1.65
Tendon injury	25	NA	0.26	NA	0.01	6.50

*2PD* Two-point Discrimination, *BCTQ-F* Boston Carpal Tunnel Questionnaire Functional Status Scale, *BCTQ-S* Boston Carpal Tunnel Questionnaire Symptom Severity Scale, *ECTR* endoscopic carpal tunnel release, *NA* not applicable, *OCTR* open carpal tunnel release, *SW* Semmes-Weinstein

^a^Heterogeneity test: I^2^ > 50%, random-effects analysis model; I^2^ < 50%, fixed-effects analysis model

^b^If odds ratio > 1, favors ECTR; if odds ratio < 1, favors OCTR

^c^If mean difference > 0, favors ECTR; if mean difference < 0, favors OCTR

The article "Open versus endoscopic carpal tunnel release: a systematic review and meta-analysis of randomized controlled trials" was published in 2020. Journal: BMC Musculoskelet Disord.

### Publication bias

Publication bias was assessed by the funnel plot method and Egger’s test. The funnel plot shape and Egger’s test (*P* = 0.869) appeared essentially symmetric (Fig. 16), indicating no overt publication bias in the analysis of complications.

**Fig. 16:** A funnel plot shows the relative symmetry in relation to the pooled estimate from the meta-analysis, indicating no overt publication bias. SE, standard error; OR, odds ratio

## Discussion

Since the development of ECTR by Chow (12) and Okutsu et al. [13] in 1989, there has been controversy regarding the superiority of ECTR over OCTR. Accordingly, many original articles have been published on this issue; moreover, several meta-analyses have compared ECTR with OCTR as treatment options for CTS [14, 15, 21–23, 55–57]. However, previous meta-analyses included fewer studies than ours, did not classify the data into subgroups according to different follow-up times, featured only a few assessments of patient outcome, and included central tendency data but not standard deviation. Therefore, we accomplished a large sample-size meta-analysis of published articles to compare the safety and effectiveness between OCTR and ECTR. The publication bias in this meta-analysis was also minimal, as demonstrated by the results of the funnel plot analysis and Egger’s test.

Our meta-analysis reviewed 28 RCTs that consisted of 2320 idiopathic CTS hands treated with two different approaches the OCTR or the ECTR. In the results it can be clearly indicated that there were no significant between-group differences in the operative time, grip strength, BCTQ-S score, BCTQ-F score, digital sensation scores, and the presence of permanent nerve injury. However, the ECTR group exhibited several clinically important advantages over the OCTR group, including higher patient satisfaction rates, greater key pinch strengths, earlier RTW times, and fewer scar-related complications.

The article "Open versus endoscopic carpal tunnel release: a systematic review and meta-analysis of randomized controlled trials" was published in 2020. Journal: BMC Musculoskelet Disord.

Consistent with the present results, previous studies demonstrated that the satisfaction rates of patients in the ECTR group were higher than those of patients in the OCTR group [24, 44, 45]. Compared with the standard open approach, generally small incisions decrease scar tenderness, reduced scarring, mild wound-related complications [53], and improvements in the major functional outcomes (key pinch strength, activities of daily living, and RTW) [31] after endoscopic release is plausible. However, it should be noted that when assessing the patient satisfaction rates, a portion of the data published by Zhang et al. [53] exhibited high heterogeneity. Therefore, these data were excluded from the present meta-analysis. The high heterogeneity was mainly because of the fact that the data compared mini-incisions with endoscopic incisions. Mini-incisions are not directly comparable to the standard incisions in OCTR, as they yield a better appearance and tend to have fewer wound-related complications than standard incisions [58].

Herein, the key pinch strength of patients was significantly greater in the ECTR group than that in the OCTR group at 3 months postoperatively [9, 31]. Additionally, previous studies reported that OCTR was associated with considerable morbidity, including increased and prolonged scar tenderness [11]. Furthermore, other studies revealed that patients who underwent ECTR experienced fewer limitations in their ability to perform daily life activities than did patients who underwent an open technique [30, 59–61]. Michelotti et al. [44] reported early differences in grip and pinch strength after ECTR; however, data were lost as the follow-up duration increased. Further studies should include a more uniform follow-up duration, and additional controlled studies with longer follow-up durations are required to clarify the effects of each technique on activities of daily living.

The finding of our meta-analysis of RCTs suggest that compared to patients treated with OCTR, those who treated with ECTR returned to work or daily activities earlier. Consistent with our results, Vasiliadis et al. [22] and Paryavi et al. [56] reported that patients who underwent ECTR experienced less surgical trauma than those who underwent an open technique, and this resulted in less time off work, faster recovery, and better performance of daily activities. However, regarding the RTW data, we noticed that divergences between the studies had large heterogeneity. A possible explanation for this large heterogeneity is that the work flexibility and the nature of the work and daily activities may have been different to a great extend in the included studies. Furthermore, while Sanati et al. [57] demonstrated the minimally invasive techniques have a great superiority over conventional open release in terms of recovery time, they highlighted the remarkable variability in how RTW as an outcome measure was examined across studies. Nevertheless, the effects of such inconsistencies were rather small when only RCTs were considered, similar to that observed in our study. Patients undergoing endoscopic release can return to work and their daily activities sooner when compared with open release.

The article "Open versus endoscopic carpal tunnel release: a systematic review and meta-analysis of randomized controlled trials" was published in 2020. Journal: BMC Musculoskelet Disord.

Our meta-analysis revealed that lower scar-related complication rates and better healing were achieved in the ECTR group while compared to the OCTR group. This may be because of the long palmar incision made during OCTR that may prolong the immobilization time and augment postoperative pain and the risk for hypertrophic or hypersensitive scar formation [22]. In contrast, ECTR uses a small incision and divides the transverse carpal ligament from below, thereby preserving the overlying skin and muscle and resulting in fewer minor complications [62, 63], particularly those related to cutaneous scars. However, previous studies demonstrated that ECTR is associated with more nerve injury; therefore, the technique is less favorable owing to its higher risk of the cutaneous branch of the median nerve iatrogenic injury [15, 19, 53]. Contrary to expectations, our study did not find a significant difference in the occurrence of permanent nerve injury between the two surgical approaches; furthermore, most noted nerve injuries were transient, and patients still achieved full recovery after surgery [29, 38, 48, 49]. Moreover, Martin et al. [64] developed a novel endoscopic system which may avoid the transient nerve injury occurring with other ECTR methods.

### Limitations

This research had two limitations. Firstly, subgroup analyses of the various ECTR techniques (one-portal and two-portal techniques) and OCTR techniques (mini-incision and long incision) were not performed. Use of different techniques may be associated with different outcomes, however, restricted by the rather limited studies and available data we were unable to divide the patients into subgroup to perform analyses. Secondly, though we included only RCTs, methodological flaws still exist, including unblinded assessments of outcomes.

Nevertheless, our study is novel since it includes the largest number of RCTs to compare ECTR and OCTR techniques. Furthermore, this is the first study to group results into different follow-up times and assess different patient outcomes, thus making the data more comparable. This study is also the first to demonstrate that ECTR is associated with better patient outcomes; we found that after careful manipulation during endoscopic surgery, ECTR can substitute OCTR.

The article "Open versus endoscopic carpal tunnel release: a systematic review and meta-analysis of randomized controlled trials" was published in 2020. Journal: BMC Musculoskelet Disord.

## Conclusions

The present meta-analysis determined that ECTR was superior to OCTR in terms of higher satisfaction rates, improved key pinch strengths, earlier RTW times, and fewer scar-related complications. Our findings suggest that patients with CTS can be effectively managed with ECTR; however, the possibility of transient nerve injury should be considered.

## Data Availability

The datasets used and/or analyzed during the current study are available from the corresponding author on reasonable request.

## Abbreviations

CTS: Carpal tunnel syndrome
OCTR: Open carpal tunnel release
ECTR: Endoscopic carpal tunnel release
RCT: Randomized controlled trial
PRISMA: Preferred Reporting Items for Systematic Reviews and Meta-Analyses
BCTQ-S: Boston Carpal Tunnel Questionnaire Symptom Severity Scale
BCTQ-F: Boston Carpal Tunnel Questionnaire Functional Status Scale
RTW: Return to work
GRADE: Grading of Recommendations Assessment, Development, and Evaluation
MD: Mean difference
CI: Confidence interval
OR: Odds ratio
SE: Standard error
